The article "Development and Application of a Standardized Testset for an Artificial Intelligence Medical Device Intended for the Computer-Aided Diagnosis of Diabetic Retinopathy" was published in 2023. Journal: J Healthc Eng.

# Development and Application of a Standardized Testset for an Artificial Intelligence Medical Device Intended for the Computer-Aided Diagnosis of Diabetic Retinopathy

**DOI:** 10.1155/2023/7139560

**Published:** 2023-02-08

**Authors:** Hao Wang, Xiangfeng Meng, Qiaohong Tang, Ye Hao, Yan Luo, Jiage Li

**Affiliations:** ^1^Institute for Medical Device Control, National Institutes for Food and Drug Control, 31 Huatuo Rd, Beijing 102629, China; ^2^State Key Laboratory of Ophthalmology, Image Reading Center, Zhongshan Ophthalmic Center, Sun Yat-Sen University, No. 54 Xianlie South Road, Yuexiu District, Guangzhou 510060, Guangdong, China

## Abstract

**Objective:**

To explore a centralized approach to build test sets and assess the performance of an artificial intelligence medical device (AIMD) which is intended for computer-aided diagnosis of diabetic retinopathy (DR).

**Method:**

A framework was proposed to conduct data collection, data curation, and annotation. Deidentified colour fundus photographs were collected from 11 partner hospitals with raw labels. Photographs with sensitive information or authenticity issues were excluded during vetting. A team of annotators was recruited through qualification examinations and trained. The annotation process included three steps: initial annotation, review, and arbitration. The annotated data then composed a standardized test set, which was further imported to algorithms under test (AUT) from different developers. The algorithm outputs were compared with the final annotation results (reference standard).

**Result:**

The test set consists of 6327 digital colour fundus photographs. The final labels include 5 stages of DR and non-DR, as well as other ocular diseases and photographs with unacceptable quality. The Fleiss Kappa was 0.75 among the annotators. The Cohen's kappa between raw labels and final labels is 0.5. Using this test set, five AUTs were tested and compared quantitatively. The metrics include accuracy, sensitivity, and specificity. The AUTs showed inhomogeneous capabilities to classify different types of fundus photographs.

**Conclusions:**

This article demonstrated a workflow to build standardized test sets and conduct algorithm testing of the AIMD for computer-aided diagnosis of diabetic retinopathy. It may provide a reference to develop technical standards that promote product verification and quality control, improving the comparability of products.

## 1. Introduction

As an emerging branch of the medical device, the AIMD, along with increasing applications of deep learning [1, 2], has demonstrated significant potential in medical imaging, image reconstruction, and postprocessing [3–16]. While hundreds of AIMDs have been approved [17, 18], the verification and validation of such devices are mainly conducted by manufacturers spontaneously, leading to variation in evaluation metrics and data sets [19]. Stakeholders show rising concern on the quality of the AIMD, such as its comparability [20] and transparency [21], which poses considerable challenges to regulation compared to a conventional medical device. In the past several years, special guidelines for the AIMD have been published [22, 23]. There are increasing efforts to establish standards for the AIMD [24–27]. The topics include terminology, performance testing, dataset quality management, and quality systems.

To support standard development, it would be helpful to explore the approach to build and apply standardized test sets. While the literature reports existing public datasets for medical AI [28, 29], they are more appropriate for model training or competition [5, 8] rather than testing. On the one hand, the design of public datasets usually occurs before the research and development of the AIMD, and they may not match the application scenario of the AIMD. On the other hand, test sets have special requirements. They should be independent from manufacturers or developers in order to verify the generalizability of AI. The capacity and diversity of data samples should be similar to the intended patient population. Standard operation protocols should be followed during the lifecycle. A systematic annotation process is needed to provide the reference standard.

This article demonstrates a case study to build test sets for computer-assisted diagnosis of DR, which is a common application of the AIMD. It is reported that deep learning algorithms can differentiate referrable DR patients from nonreferrable DR patients by reading colour fundus photographs [5, 7, 9, 10, 12]. Indeed, annual DR screening using digital photographs of the retina has long been recommended by several major governmental or professional organizations, including the UK National Health Service [10, 30], the American Diabetes Association [31], and other international societies [32].

In this article, a standardized approach is proposed to compose test sets for DR. The major procedure is described, including data collection, curation, and annotation. The test set is applied in the testing of AUTs. The advantages and practical issues of this approach are discussed, which may provide a reference for the development of technical standards.

## 2. Materials and Methods

### 2.1. Framework for Dataset Construction

The framework to build the test set is illustrated in Figure 1. It depicts a workflow, including design input, requirement specification, data collection, data curation, data annotation, and quality inspection. Risk management and personnel management are also considered and integrated into the workflow.

### 2.2. Design Input and Requirement Specification

To initiate dataset construction, the design input is firstly clarified. The intended use of this test set is to verify algorithm performance on classification of diabetic retinopathy by comparing algorithm outputs with the reference standard. The test set represents colored fundus photographs of diabetic patients from hospitals. Common image formats such as JPEG and BMP are accepted.

Requirement specification of this test set further describes dataset composition, classification, and data inclusion/exclusion criteria. This study uses colored photographs taken by fundus cameras that are officially approved to enter the market with a field of view no less than 45°. Photographs taken under near-infrared illumination are not included. According to the common intended use of AIMD products and the clinical guidelines for DR [33, 34], the images in the test set should include 7 categories (shown in Table 1): no apparent DR, mild nonproliferative DR (NPDR), moderate NPDR, severe NPDR, proliferative DR (PDR), other fundus diseases, and ungradable images (low image quality). No apparent DR and mile NPDR are considered nonreferrable. Moderate NPDR, severe NPDR, and PDR are considered referrable. The proportion of referrable DR in the test set should be similar to the prevalence in the patient population.

Notably, the above categorization method is a result of justification since many AI products in China were designed according to the Guidelines for Diabetic Retinopathy Diagnosis and Treatment in China [33], which has referenced a previous version of the guidelines published in 1985 and ICO guidelines for diabetic eye care. The current guideline [33] divides DR based on severity into 6 stages as shown in Table 2. DR phases 0–III in Table 2 are equivalent to Classes 0–3 in Table 1. Since the treatment scheme of DR phases IV–VI is similar and the referral strategy is identical, the test set consolidates these stages into Class 4, which is compatible with ICO guidelines and practical in a clinical scenario.

Fundus diseases other than DR are classified as Class 5, which include but are not limited to hypertensive retinopathy [35], age-related macular degeneration [36], suspect glaucoma [37, 38], retinal vein occlusion [39], pathologic myopia [40], and optic nerve diseases [41]. Although these ocular diseases are not necessarily claimed by AIMD products, they may be imported into AIMDs in the real world. Therefore, they serve as negative controls in the test set.

Ungradable images are classified as Class 6. Image quality is given special attention in the development of the test set. DR screening is often performed in out-patients, sometimes on patients with undilated pupils. The colour retinal photographs are obtained using low levels of illumination. Also, human factors such as movement and positioning in addition to ocular factors such as cataracts and reflections from retinal tissues can produce defects. Especially, without pupillary dilatation, artifacts are observed in 3–30% of retinal images to the extent that they impede annotation [42]. Therefore, in this test set, ungradable images are also included, with conditions ranging from over darkness/saturation, out of focus, wrong positioning, lens contamination, to anterior segment images.

If an image only has minor quality problems that do not disturb annotation, it will be annotated and assigned to category 0–5. Images with photocoagulation marks and other treatment marks are annotated according to their posttreatment features. The comparison between pretreatment and posttreatment images is not within the scope of the test set.

### 2.3. Risk Management

Data security, patient privacy, and data bias are the major risks considered in this study. To ensure data security, all activities are conducted on the local area network with controlled user access. Data are stored in servers independent from algorithms under testing. Data annotation tools are not allowed to export images. To protect patient privacy, only deidentified images with ethical approval are accepted in this test set. To minimize data biases such as selection bias and coverage bias, the diversity of positive and negative samples is highlighted in the requirement specification.

### 2.4. Data Collection

During data acquisition, deidentified fundus photographs are collected retrospectively from partner hospitals with ethical approval from local institutional review boards. The raw images are submitted in JPEG formats. No modification or processing, such as filtering, smoothing, clipping, and contrast enhancing, is allowed. Additional information on image sources, including data collection sites, manufacturers of fundus cameras, and models of fundus cameras, is recommended and submitted.

### 2.5. Data Curation

Data curation is the process to ensure data safety and quality. First, the status of deidentification and ethical approval proof are manually confirmed. Second, data vetting is conducted to exclude problematic images, including unreadable files, incomplete images, and images that compromise privacy information. After curation, the images are stored, indexed, and submitted to the image annotation process. Additional data preprocessing is not implemented in this study.

### 2.6. Resource Management

Dataset construction relies on resource management, especially personnel management and tool management.

Personnel management focuses on annotator recruitment, qualification, and management. The annotation task needs both junior annotators and senior annotators. All junior annotator candidates are publicly recruited. The basic qualification is a board-certified ophthalmologist with at least 5 years of clinical experience. All candidates receive annotation instructions in advance to clarify the classification rule according to the literature on DR [33, 34] and other fundus diseases [35–41]. After the training, the candidates attend an exam to classify 100 fundus photographs (18% nonreferrable DR, 45% referable DR, 32% other ocular diseases, and 6% ungradable images). Those who achieve greater than 80% accuracy pass the exam. They are given an additional training session.

Senior annotators should have professional certification as image readers and receive special training to promote consistency. In this article, senior annotators all have NHS (UK National Health Service) certification.

Tool management focuses on software tools that facilitate data processing and annotation. In this study, a custom-built annotation software is used. The main functions include image preview, contrast adjustment, image magnification, filter selection, task assignment, and progress monitoring. Annotators can add, edit, and submit annotation results. Reviewers and arbitrators can visit their results and make corrections or justifications. The software only exports annotation results. No modifications are made to images.

### 2.7. Data Annotation

The reference standard is based on the combined decisions of junior annotators and arbitration experts. The image annotation is conducted in a laboratory environment. The annotation workflow is summarized in Figure 2. The annotation process includes two rounds:

#### 2.7.1. First Round (Initial Annotation)

Each batch of images is assigned to a team of 3 annotators. The annotators independently annotate images in a blinded way. If their classification result on an image is fully in agreement, such images are categorized as the prequalified pool. Images with discordant classifications are categorized as the arbitration pool. 10% of the prequalified pool is randomly sampled and submitted to the second round. The annotations of the rest of the prequalified pool are accepted conditionally. The arbitration candidate group are also submitted to the second round.

#### 2.7.2. Second Round (Review and Arbitration)

This step is carried out by a team of three senior annotators, one of whom acts as the team leader. The team leader has served as the director of an image reading center in a top ophthalmological hospital. They review all images submitted to this round so as to resolve the final annotation in the arbitration pool and review the samples from the prequalified pool. If sampled annotation results in the prequalified pool cannot pass the review, more samples will be submitted to the arbitration pool. Feedback may be given to annotators in the first round. Senior experts can justify the number of samples in the prequalified pool for inspection.

All images are stored, accessed, previewed, and manually classified using a custom-built annotation software.

### 2.8. Quality Inspection

After data annotation, quality inspection is conducted to examine the dataset's quality. The annotation records, including initial annotation, review, and arbitration, are reviewed and compared on each image to avoid inconsistencies and mistakes. Images that pass quality inspection are enrolled in the test set. The percentage of diabetic retinopathy subtypes is calculated. Usability and validity of each image are also examined manually.

### 2.9. Algorithm Testing

Five algorithm models intended to classify fundus photographs are enrolled as AUTs. They are trained by different manufacturers or developers. They all claim to use deep learning, but details such as the neural network structure, weights, and training sets are beyond the scope of this article. The test set is imported into each AUT. The output of AUTs is compared with the final annotation results. The overall accuracy, sensitivity, and specificity used to differentiate referable DR from nonreferrable images are reported. The performance of AUTs is further compared across the 7 subtypes separately.

## 3. Results

### 3.1. Diversity of the Test Set

The test set contains 6327 images from 11 hospitals in 10 provinces. Among them, 9 hospitals are tertiary hospitals and contribute 71.2% of the images, while the rest are secondary hospitals and contribute 28.8%. No primary hospitals or community clinics are involved. Since the images are deidentified, the location of the hospital is used to indicate geological distribution of patients. The provincial distribution of images is shown in Table 3, which demonstrates that representative provinces in Northeast China, North China, Central China, East China, Southeast China, and South China are involved.

The images are acquired by more than 13 types of fundus cameras made by 9 manufacturers, all in compliance with an ISO standard on fundus cameras [43]. The field of view is 45°. The optical resolution is between 80 and 120 pairs s/mm. All images are larger than 1000 pixel by 1000 pixel. The difference in image size, detector, light source, and embedded software may add more diversity to image quality and features.

In this test set, all fundus photographs are rectangular images with a pure background (either dark or white pixels) enveloping the round-shaped images of interest. The ratio between the pure background area and the whole area of each photograph is also considered an important source of image variation.

### 3.2. Performance of Annotators

During the recruitment of annotators, 47 ophthalmologists registered and attended the exam to classify 120 fundus images, including 63 DR images. 15 candidates finally passed and joined the annotation. Their average professional experience is above ten years. They are from 15 different hospitals in 7 provinces. Their accuracies in the exam range from 80% to 87%. The interannotator agreement is evaluated by calculating Fleiss' kappa. The result is 0.75, which is considered substantial given the fact that annotators come from different hospitals and regions. The intraannotator agreement is evaluated by calculating intraclass correlation, which is >85% for all qualified ophthalmologists. Additional training is given before the centralized annotation to reinforce the guidelines and minimize misunderstandings.

### 3.3. Annotation Results

In the first round, 15 annotators are evenly divided into 5 groups randomly. Individual workload is between 1000 and 1500 images. 3694 images yield concordant results, and 369 images are submitted to the second round as samples for inspection. 2356 images are graded with a majority opinion reached within each grading group and submitted to the second round for arbitration. 277 images yield totally diverse results within each group and are sent for arbitration too.

In the second round, the images are read by two NHS certified retinal experts and a senior expert with an NHS certificate independently in a blinded way. Then, they discuss all results and reach consensus on the final annotation results. According to the final results, 55.41% of images are directlydetermined by the consensus within each group in the first round. 16.02% of the images are graded according to the major opinion within each group in the first round. 26.81% of the images are graded with a reference to the minor opinion in each group in the first round. Only 1.76% of the images are graded only by the arbitrators.

Using the final annotation results as the reference standard, the accuracy of each annotator is calculated. The average accuracy is 83%. The minimum is 75%, while the maximum is 90%. 13 out of 15 annotators have accuracy higher than 80%. The performance of the 15 annotators comports with their qualification exam results and is considered satisfactory in comparison with the commonly accepted diagnostic accuracy by single-field fundus photography [42].

The composition of the annotated images is described in Table 4. The overall proportion of DR is 39.51%, comparable with the prevalence of DR in the Chinese DM population (24.7%–37.5%) [33]. The prevalence of other fundus diseases is 41.08%. This test set balances the proportion between DR and other fundus diseases that may be assessed by future AIMD products.

The classification of the current test set can be expressed in a simplified manner. Class 0 and Class 1 in Table 1 are consolidated into nonreferrable DR. Class 2 to Class 4 in Table 1 are consolidated into referrable DR. Class 5 and Class 6 may remain independent or be consolidated into a certain type. In the following algorithm testing, they are considered nonreferrable.

### 3.4. Comparison with Raw Labels

During data collection, partner hospitals submitted raw labels, which were annotated by local annotators without centralized examination or training. The number of annotators deployed in each hospital varied from 1 to 3. The requirement for annotator qualification was different among partner hospitals. The minimum requirement was graduate student level, and the maximum requirement was associate professor level. Using the final annotation results as the reference standard, the overall accuracy of raw labels is 61.64%, and Cohen's Kappa is 0.5173, indicating the quality problems with raw labels.

### 3.5. Algorithm Testing Results

The overall accuracy, sensitivity, and specificity to differentiate referable DR from nonreferrable images are calculated and compared among the 5 AUTs.  Table 5 shows the results of the 5 AUTs. The accuracy ranges from 0.77 to 0.88. The sensitivity ranges from 0.80 to 0.86. The specificity ranges from 0.73 to 0.89. AUT1 shows the highest accuracy and sensitivity among the 5 AUTs.

The capability of the algorithm to correctly classify images of a specific class as referable or nonreferrable is also calculated. For class 2–class 4, it is represented as the number of true positives over the total number of samples in this category, which is equivalent to sensitivity. For other classes, the specificity of each category is calculated instead.  Table 6 compares the performance of 5 AUTs on each specific class. It provides more details to demonstrate the variation in algorithm performance. For class 0, class 3, and class 4, the capability of all AUTs is above 95% on average. For class 1, the capability of AUT1 is significantly lower than the rest (on average above 90%). For class 2, the capability ranges from 0.64 to 0.75, indicating a common weakness among all 5 AUTs. For class 5, the capabilities of AUT1 and AUT3 significantly outweigh the rest of the AUTs. For class 6, AUT1 shows the top capability among the 5 AUTs. No AUTs in this experiment shows homogeneous capability to classify all 7 classes.

## 4. Discussion

This article demonstrates a centralized pathway to build test sets and conduct third party testing of AIMD products. The test set is composed of 6327 images, which are annotated into 7 classes covering all stages of DR according to ICO guidelines, as well as “other fundus diseases” and “ungradable images.” The diversity of the test set considers data sources (11 hospitals from 10 provinces), fundus cameras (>13 models from 9 manufacturers), and image parameters (image sizes, detectors, and light sources).

The pathway for test set construction in this article is different from that in algorithm challenges, where test sets and training sets are usually constructed under the same protocol or as subsets of a larger dataset. This pathway relies on independent data collection, curation, annotation, and storage, which decreases the possible similarity between this test set and training sets owned by developers of AUTs and promotes the verification of AI algorithm generalizability. It may be suitable for third party testing laboratories to conduct conformity assessment.

According to the literature [5, 9, 10, 44], the pathway to form the reference standard in other studies is based on various combinations of annotators and reviewers. In this study, a combination of prequalified annotators and arbitrators conducted data annotation. Under this scheme, the annotators' performance is estimated quantitatively (Fleiss Kappa = 0.75, individual accuracy >80%, and intra-class correlation >85%). During the annotation process, each image in the test set is reviewed by 3–6 experienced professionals, and 98.2% are determined by the major decision (3 votes out of 3 annotators or >4 votes out of 6). Only 1.76% are determined by the arbitration experts. The results show that the annotation scheme helps enhance consensus among annotators.

On the other hand, the raw labels from partner hospitals show significantly lower accuracy and consistency compared to the final annotation results. According to information provided by partner hospitals, the raw labels are annotated by an inconstant number of annotators, ranging from 1 to 3, including graduate students, residents, and junior and senior ophthalmologists. It suggests the importance to organize annotation task systematically and the necessity to establish consistent annotation rules among different hospitals. Otherwise, the discrepancy in data annotation may impact dataset quality and further inhibit the quality of the AIMD.

Using the annotated test set, the performance of 5 AUTs is tested quantitatively as technical demonstration. It is straightforward to compare the overall accuracy, sensitivity, and specificity in the scenario of DR classification. Algorithm performance can be further observed on subgroups of the test set. However, no AUT in this experiment shows homogeneous capability to classify different categories of images. While public stakeholders pay attention to algorithm fairness and generalizability, this study shows the necessity to reveal and understand how the AI algorithm performs differently on subtypes of diabetic retinopathy images. It also indicates that algorithm performance may change with the proportion of these categories. A strategy to tune the composition of test sets in a flexible manner is needed to guide future testing.

This work explores practical approach and issue in advancing the standardized testing of the AIMD. But due to time and resource constraints, it has limitations in the following aspects:

First, the test set is based on retrospective data collection. Although data are randomly sampled by partner hospitals, control measures should be taken to limit bias. Continuous sampling of data within a period may help.

Second, the proportion of mild NPDR is much smaller than that of other DR subtypes. One possible reason is that without compulsory DR screening, patients with mild NPDR are unlikely to take fundus photographs, which results in the relative scarcity of mild NPDR photographs. Increment of mild NPDR not only decreases the sampling errors of SE and SP but also improves the balance between different stages of DR. In fact, from the annotator's perspective, it is important to differentiate microaneurysm in mild NPDR from blot hemorrhages in moderate NPDR. Therefore, more cases of mile NPDR should be added to the current test set.

Third, as a colour fundus photograph dataset, it is difficult to use the test set alone to annotate important diseases among the 41.09% “other diseases” that may be assessed by AI in the near future. Colour fundus photographs are incapable of thickness measurement, which inhibits detection of certain diseases such as AMD and glaucoma. Images from additional imaging modalities such as OCT should be added to the test, but the cost will increase significantly.

Fourth, the diversity of this test set still needs improvement. Partner hospitals in this study are mostly tertiary hospitals, without community-level hospitals. As a result, most photographs are acquired by high-end fundus cameras. Handheld fundus cameras, which may be more popular in community-level clinics and rural areas, have minor contribution to data collection. More data should be added to compensate for this scenario and enrich data diversity.

To promote standardization of AIMD testing, reliability and comparability of test sets need to be addressed in the future research. Test sets built by different organizations may have different data sources, data inclusion/exclusion criteria, annotation resources, and procedures, which would cause inconsistent dataset quality. Transparent description of data sets should be normalized. Consensus standards on dataset construction and annotation are needed to guide the procedure. It would be necessary to conduct sample inspection and comparison among test sets, similar to proficiency testing [45] by interlaboratory comparison.

## 5. Conclusions

This article proposes a practical approach to build test sets for third-party testing of the AIMD. It takes quality control measure during data collection, curation, and annotation. It demonstrates the benefit of centralized data annotation in comparison with individual annotators and spontaneous annotation from single hospitals. The application of such a test set reveals algorithm performance and weakness in a comparative and straightforward manner, providing helpful information for regulation of such medical devices.

## Figures and Tables

**Figure 1:** standardized framework for dataset construction.

**Figure 2:** The annotation workflow.

**Table 1:** The categorization of the test set.

Class	Meaning
0	No apparent DR
1	Mild NPDR
2	Moderate NPDR
3	Severe NPDR
4	PDR
5	Other fundus diseases
6	Ungradable images

**Table 2:** Definition of DR phases.

DR phases and findings observable on fundus photos [33]	Classes in ICO guidelines [32]
0: no abnormalities	No apparent DR

I: microaneurysms only	Mild NPDR

II: microaneurysms and other signs (e.g., dot and blot hemorrhages, hard exudates, and cotton wool spots), but less than severe nonproliferative DR	Moderate NPDR

III: moderate nonproliferative DR with any of the following:	Severe NPDR
(1) Intraretinal hemorrhages (≥20 in each quadrant)	
(2) De nite venous beading (in 2 quadrants)	
(3) Intraretinal microvascular abnormalities (in 1 quadrant)	
(4) No signs of proliferative retinopathy	

IV: neovascularization of the optic disc or elsewhere. When accompanied by vitreous/preretinal hemorrhage, it is defined as high risk PDR	Proliferative DR (PDR)
V: fibrous membrane could be accompanied by preretinal hemorrhage or vitreous hemorrhage	
VI: traction retinal detachment, combined with fibrous membrane, combined with/without vitreous hemorrhage, and neovascularization of the iris and the anterior chamber angle	

**Table 3:** Geological distribution of image sources.

Region	Province	Percentage
North China	Beijing	16

Northeast China	Heilongjiang	13
	Liaoning	22

Central China	Henan	2
	Hubei	2

East China	Shanghai	9
	Zhejiang	4
	Anhui	3

Southeast China	Fujian	15

South China	Guangdong	14

Total		100

**Table 4:** The distribution of annotated images.

Class	Number	Percentage
0: no apparent DR	873	13.798
1: mild NPDR	262	4.141
2: moderate NPDR	1118	17.670
3: severe NPDR	579	9.151
4: PDR	540	8.535
5: other fundus diseases	2600	41.094
6: ungradable	355	5.611
Total	6327	100

**Table 5:** Comparison of overall performance metrics.

Metrics	AUT1	AUT2	AUT3	AUT4	AUT5
Sensitivity	0.861422	0.814484	0.831024	0.802861	0.851587
Specificity	0.884597	0.820782	0.890465	0.799267	0.728851
Accuracy	0.876403	0.818555	0.869448	0.800537	0.772246

**Table 6:** Comparison of decision capability among 5 AUTs.

Class	AUT1	AUT2	AUT3	AUT4	AUT5
0	0.983963	0.989691	0.988545	0.988545	0.934708
1	0.557252	0.958015	0.912214	0.885496	0.889313
2	0.752236	0.645796	0.677102	0.639534	0.746869
3	0.982729	0.991364	0.993092	0.984455	0.977547
4	0.957407	0.974074	0.975926	0.946296	0.933333
5	0.893846	0.801923	0.889231	0.761153	0.642308
6	0.814085	0.442254	0.642254	0.549295	0.738028

## Data Availability

The data supporting the findings of the current study are available from the corresponding author upon request.
